# Depression, anxiety and associated factors among people with epilepsy and attending outpatient treatment at primary public hospitals in northwest Ethiopia: A multicenter cross-sectional study

**DOI:** 10.1371/journal.pone.0256236

**Published:** 2021-08-13

**Authors:** Kabtamu Nigussie, Alemu Lemma, Addisu Sertsu, Henock Asfaw, Habtamu Kerebih, Tilahun Abdeta

**Affiliations:** 1 Department of Psychiatry, School of Nursing and Midwifery, College of Health and Medical Sciences, Haramaya University, Harar, Ethiopia; 2 Department of Psychiatry, School of Medicine, College of Medial and Health Sciences, University of Gondar, Gondar, Ethiopia; 3 Department of Nursing, School of Nursing and Midwifery, College of Health and Medical Sciences, Haramaya University, Harar, Ethiopia; UCSI University, MALAYSIA

## Abstract

**Objective:**

To assess the magnitude and factors associated with depression and anxiety among people with epilepsy and attending out-patient treatment at central Gondar zone primary public hospitals, northwest, Ethiopia.

**Method:**

An institutional based cross-sectional study was conducted from May—June, 2020 at central Gondar zone primary public hospitals. A total of 589 participants were chosen by systematic sampling technique. Data was collected by utilizing Amharic version interviewer-administered structured and semi-structured questioners. Depression and anxiety were assessed by using hospital anxiety and depression scale. Bivariate and multivariate logistic regression analysis was done to recognize variables related to both depression and anxiety. Association was described by using “adjusted odds ratio” (AOR) along with 95% full Confidence interval (CI). Finally, P-values < 0.05 in adjusted analysis were taken as a cut off for significant association.

**Result:**

Out of 556 participants included in the study, 30.9%, 33.1% had depression and anxiety respectively. Being divorced/widowed (AOR = 2.43, 95% CI, 1.18–4.99), using two and above number of antiepileptic medications (AOR = 1.77,95% CI,1.02–3.09), very frequent seizure frequency (AOR = 2.68, 95% CI,1.30–5.51), current substance use (AOR = 1.82, 95% CI, 1.03–3.22), perceived stigma (AOR = 5.67,95% CI,3.14–8.18), and hazardous alcohol use (AOR = 2.84, 95% CI,1.32–6.09) were statistically associated with depression. While, being a single (AOR = 1.65, 95% CI, 1.04–2.63), using two and above number of antiepileptic medications (AOR = 2.27, 95% CI, 1.42–3.62), duration of illness ≥16 years (AOR = 2.82, 95% CI, 1.26–6.31), and perceived stigma (AOR = 2.49, 95% CI, 1.63–3.82) were statistically associated with anxiety at a p-value < 0.05.

**Conclusion:**

This study showed that the magnitude of depression and anxiety were relatively high among people with epilepsy. Using two and above number of antiepileptic medications and perceived stigma were statistically associated with both depression and anxiety. Screening, early identification and providing appropriate intervention of depression and anxiety among people with epilepsy should be great concern for the health care providers.

## Introduction

Epilepsy is a neurological condition involving the brain that produces individuals more vulnerable to having repetitive, ridiculous seizure, which has brief scenes of involuntary movement that may involve a part of the body (partial) or the entire body (generalized) and are sometimes accompanied by loss of consciousness and control of bowel or bladder function [1, 2]. It affects around 50 million individuals around the world, making it one of the foremost common neurological diseases universally [2].

According to report of World Health Organization (WHO) about 80 percent of individuals with epilepsy live in low- and middle-income nations and it is estimated that up to 70 percent of people living with epilepsy seem live seizure- free in case appropriately analyzed and treated. The risk of untimely passing in people with epilepsy is up to three times higher than for the general population [2].

Depression is disruption of mood characterized by loss of interest, discouraged temperament, unsettling influence of sleep, problem in appetite and psychomotor action, trouble to concentrate or make decision, blameworthy or evil feeling, easily tiredness and repeating considerations of death or suicide [3]. Anxiety is also the presence of fear or trepidation that’s out of extent to the setting of the life circumstance and it can be expressed in several ways such as uncontrollable stress, strongly fear, upsetting dreams or flashbacks of a traumatic event [4].

Depression is the most common type of psychiatric co-morbidity in people with epilepsy. It is more likely to happen in patients with partial seizure disorders of transient (temporal) and frontal lobe origin and are more frequent among patients with ineffectively controlled seizures [5]. Depression can directly increase seizure recurrence through the mechanism of sleep deprivation; disappointment to recognize sadness or lacking treatment can lead to suicide [6]. Anxiety can be indeed more common, occurring in around 25 percent of people with epilepsy in a community setting though in secondary care and specialist centers its predominance surpasses 50 percent [7].

Different studies across the world showed that there is high magnitude of depression and anxiety among people with epilepsy with prevalence rates ranging from 20% to 55% [8]. The prevalence of depression and anxiety in UAE was reported (26.9% and 25.8%), in China (52.6% and 33.4%), in Brazil (24.4% and 39.4%), and in Thailand (20% and 39%) respectively [8–11]. Study in sub -Saharan Africa revealed that range prevalence of depression and anxiety among people with epilepsy were 39.4%-49.3% [12–16] and 33.1%-47% of respectively [17–19].

On the other hand, different variables were reported as having a significant association with depression and anxiety disorder among individuals with epilepsy. Female sexual orientation, frequent seizures, perceived stigma, suicidality, poly treatment and destitute seizure control were risk factors for anxiety disorders [9, 11, 18, 20]. On other hand, male gender, being married, low socio-economic status, uncontrolled seizure and poly therapy, having frequent seizure frequency, head trauma, perceived stigma, lower educational level and suicidality were significantly associated with depression [11, 20, 21].

However, there is a deficiency of enough epidemiological data on depression and anxiety among people with epilepsy in Ethiopia. Therefore, this study was aimed to assess the prevalence and correlated factors of depression and anxiety among people with epilepsy attending out-patient treatment at primary public hospitals in northern part of Ethiopia.

## Materials and methods

### Study setting

This study was conducted during the period from May to June, 2020, at central Gondar zone among randomly selected four primary public hospitals which are Wogera, Dembia, Delagi and Aykel primary hospitals. Central Gondar zone is located in Amhara regional state, northwest part of Ethiopia and there are 8 primary public hospitals in this zone which give service to around 2.5 million people.

### Study design

Institutional based cross-sectional study design was conducted.

### Source population

All people with epilepsy who visit central Gondar zone primary public hospitals.

### Study population

All adults aged ≥ 18 years, who had been clinically diagnosed with epilepsy and who attended out-patient treatment service at Wogera, Dembia, Delagi and Aykel primary hospitals during the study period were study participants. Individuals who were unable to communicate and seriously ill at the time of the data collection period were excluded.

### Sample size determination and sampling technique

The adequate sample size was calculated by using a single population proportion formula(n = (Zα/2)2 p (1-p)/ d2) with assumption of, a 33.5% prevalence of depression [22], 4% tolerable margin of error, 95% confidence interval with 10% non-response rate. Therefore a minimum 589 number of participants were required to conduct this study. A systematic random sampling method with the sampling fraction of 2 was used to select study participants from the selected primary public hospitals during the study period. Sampling interval was determined by dividing the total study population who to follow up during the data collection period approximately 1192 by total sample size 589.The sampling fraction or k = x/y = 1192/589 = 2.02≈2. The first study participant was selected by a lottery method from each hospital independently, and the next study participants were selected at a regular interval (every 2) individual as shown in (**Fig 1)**.

**Fig 1:** Schematic presentation of sampling procedure for assessment of magnitude and associated factors of depression and anxiety among people with epilepsy at out-patients treatment at central Gondar zone public hospitals, northern part Ethiopia.

### Data collection tools and technique

Hospital anxiety and depression scale (HADS) were used to assess depression and anxiety. Hospital anxiety and depression scale was used and validated in Ethiopia with internal consistence of 0.78, for anxiety sub-scale 0.76, for depression sub-scale and 0.87 for the full hospital anxiety and depression scale. It is commonly used to screen anxiety and depression symptoms and it has 14 item questions which are divided into two parts, which is a 7- item sub-scale for each depression and anxiety symptoms. The items are rated on a four-point Likert scale which is ranging from 0 to 3 giving maximum and minimum score of 0 and 21 receptively. If the participants scores ≥8 for each depression and anxiety sub-scale questions were considered as the participant has anxiety and depression respectively [23]. The internal consistency by Cronbach’s alpha of hospital anxiety and depression scale in this study was 0.84, 0.82, for depression and anxiety respectively.

Hazardous alcohol use was assessed by Fast Alcohol Screening Test, which was a 4-items brief screening questionnaire. FAST (Fast Alcohol Screening Test), was extracted from AUDIT (alcohol use disorder identification test) which used to measures hazardous alcohol use. FAST five different item questions, each item was scored from 1 to 4, whose total score was considered weather the participants has as hazardous alcohol use or not hazardous alcohol use. A mean score of ≥3 was indicated hazardous alcohol use [24]. It was utilized to think about alcohol used within the east-Africa setting, including Ethiopia [25]. FAST was illustrated with sensitivity of 91% and specificity of 93% [24]. The FAST internal consistency in Cronbach’s alpha of this study was 0.81.

Social support was assessed by Oslo-3 item of social support scale. It is 3 item questionnaires, commonly used to assess social support and it has been used in several studies. The sum score scale ranging from 3–14, which had three categories: poor support 3–8, moderate support 9–11 and strong support 12–14 [26]. The internal consistency, Cronbach’s alpha of Olso-3 items in the current study was 0.85.

Perceived stigma was assessed by kilifi stigma scale (KSS) which was developed and validated in kilifi, Kenya, with high internal consistency Cronbach’s alpha of 0.91 and excellent test- retest reliability with gamma 0.92. It is a simple three-point likert scoring system scored as not at all (0), sometimes (1) and always (2). A total of score was calculated by adding of all item scores. A patient who score above 66th percentile of the data measured by kilifi stigma scale of epilepsy indicate presence of perceived stigma [27]. The Cronbach’s alpha, of kilifi stigma scale in the current study was 0.94.

Data were collected by face-to-face interviews using Amharic version a semi-structured and structured interviewer administered questionnaire and manually reviewing the patient chart by six trained bachelors of Science in psychiatric nurse. The data collection process was supervised by 2 trained supervisors who had MSc in public health.

### Data processing and analysis

The data was checked for completeness, consistency and entered to Epi-Data version 4.6.0.2 and was exported to SPSS (Statistical Package for Social Science) version 20 for analysis. Bivariate and multivariate logistic regression analysis was performed to identify factors associated with outcome variable. All variables with a p-value less than 0.25 in bivariate analysis were entered into the multivariate logistic regression analysis. A p-value of < 0.05 was considered as statistically significant, and the adjusted odds ratio (AOR) with 95% confidence interval (CI) was calculated. Goodness of model fitness was checked by using Hosmer-lemshow test.

### Data quality control

The questionnaire was translated to the Amharic language to be understandable by all participants and re-translated back to English to ensure its consistency. One day training was given to data collectors about ethical principle, confidentiality, how to interview and data management. Pretest was done on 5% of the final sample size at the university of Gondar comprehensive specialized hospital. The result was not included in the result of this study finding. Based on the finding of the pretest data, the questionnaire was checked for its clarity, simplicity, and understandability. The data collectors were supervised daily, and the field questionnaires were checked daily for completeness by the supervisors and the principal investigator.

### Ethical consideration

Ethical approval was obtained from the Ethical review board of the University of Gondar, college of medicine and health science, Institutional Health Research Ethics Review Committee with a reference number (IHRERC/083/2020). A formal permission letter was obtained from school of medicine, University of Gondar and it was taken to selected hospitals which are, Delagi, Wogera, Dembia, Aykel primary hospitals. Participants were informed about the aim of the study and the advantage of the study; confidentiality, there was no any risk of being participants, and they have full rights to halt in the middle of the interview. Oral informed consent was taken from each participant before data collection takes began.

## Results

### Socio-demographic characteristics of the study participants

Out of a total 589 samples, 556 participants were included in the study with response rate of 94.4%. The median age of respondents was 31 with an interquartile range of (IQR, 24–38) years. The large part of participant 57.6% (320) were males. With respect to living condition of participants, 66.2% (368) were living with family. Around two third of them, 62.9% (367) were orthodox Christian religious followers and 34. % (189) was farmers as show below in (**Table 1**).

**Table 1:** Socio-demographic and economic distributions of people with epilepsy at central Gondar zone primary public hospitals, northern part Ethiopia (n = 556).

Variables	Categories	Frequency(n = 556)	Percentage (%)
**Sex**	Male	320	57.6
	Female	236	42.4
**Age in years**	18–24	167	30.0
	25–31	195	35.1
	32–38	83	14.9
	39–45	57	10.3
	>45	54	9.7
**Marital status**	Single	202	36.3
	Married	284	51.1
	Divorced/widowed	70	12.6
**Living condition**	With family	368	66.2
	Alone	188	33.8
**Religion**	Orthodox	350	62.9
	Muslim	127	22.8
	Protestant/catholic	79	14.2
**Occupation**	Government worker	53	9.5
	Merchant	118	21.2
	Framer	189	34.0
	Student	62	11.2
	Unemployed	81	14.6
	Household worker	53	9.5
**Education**	No formal education	117	21.0
	Primary (1–8)	240	43.2
	Secondary (9–12)	135	24.3
	Tertiary and above	64	11.5
** Residence**	Rural	344	61.9
	Urban	212	38.1
**Monthly income In Ethiopian birr**	≤550	145	26.1
	551–1000	174	31.3
	1001–2124	103	18.5
	>2124	134	24.1

1(one) Ethiopian Birr = 0.023 US dollar.

### Clinical, psychosocial, and substance related factors of participants

Around two-third, 68.2% (379) of respondents reported the age onset of epilepsy when they were ≥ eighty years and above. About half 44.0% (248) of respondents had one to six years duration of treatment whereas 45.3% (252) had up to five years duration of illness. Greater than ¾(three-fourth), 79.0% (439) of respondents were taking 1 anti-epileptic medication. From all study respondents 10.1% (57), and 10.3% (58) had family history of mental illness and family history of epilepsy respectively whereas 8.6% (49) had history of other medical illness. With respect to social support nearly two-third, 66% (367) had moderate social support. From all study respondents, 66.7% (371) and 27.9% (155) had no perceived stigma and current substance users respectively as shown below in (**Table 2**).

**Table 2:** Description of clinical, substance use, psychosocial features of people with epilepsy at central Gondar zone primary public hospitals, northern part of Ethiopia (n = 556).

Variables	Categories	Frequency(n = 556)	Percentage (%)
Age onset of epilepsy	<18 years	177	31.8
	≥18 years	379	68.2
Duration of treatment (years)	Up to 1	115	20.0
	1–6	252	45.3
	7–12	142	25.7
	>12	46	8.3
Duration of illness(years)	Up to 5 years	349	62.8
	6–10 years	121	21.8
	11–15 years	55	9.9
	16 years and above	31	5.6
Number medication	One	439	79.0
	Two and above	117	21.0
Types of medication	Phenobarbitone	318	57.2
	Phenytoin	130	23.4
	Na valproate	85	15.3
	Carbamazepine	23	4.1
Frequency of seizure	Very frequent	92	16.5
	Frequent	152	27.3
	Occasional	199	35.8
	Rare	113	20.3
Other medical illness	Yes	48	8.6
	No	508	91.4
Any family members with of mental disorders	Yes	57	10.1
	No	506	89.9
Family history of epilepsy	Yes	58	10.3
	No	505	89.7
Any Medication for other mental disorders	Yes	87	15.6
	No	469	84.4
Social support	Poor	111	20
	Moderate	367	66
	Strong	78	14
Perceived stigma	Yes	185	33.3
	No	371	66.7
Ever substance use	Yes	230	41.4
	No	326	58.6
Current substance use	Yes	155	27.9
	No	401	72.1
Hazardous alcohol use	Yes	79	14.2
	No	477	85.6

### Factors associated with depression among people with epilepsy

In crude (bivariate) logistic regression analysis variables like living alone, being single, divorced/widowed, being unemployed, taking two and above antiepileptic medications, experiencing antiepileptic medication side effects, very frequent seizure frequency, current substance use, perceived stigma and hazardous alcohol use were significantly associated with depression. However, in the multivariate logistic regression analysis variables like being divorced/widowed, taking two and above anti-epileptic medications, very frequent seizure frequency, current substance, perceived stigma, and hazardous alcohol use were statistically significantly associated with depression with p-value less than 0.05.

In this study, the odds of having depression among participants with being divorced/widowed was about 2.43 times higher as compared to participants those being married (AOR = 2.43, (1.18–4.99)) and the odds of having depression among respondents who had took two and above anti-epileptic medications was 1.77 times higher as compared to respondents who had took only one anti-epileptic medication (AOR = 1.77, (1.02–3.09)).

The odds of having depression among participants who had very frequent seizure frequency was 2.68 times higher as compared to participants who had a seizure frequency occurring at interval longer than one year (AOR = 2.68, (1.30–5.15)).

The results of this study showed that the odds of having depression among participants who had perceived stigma was about 5.07 times higher as compared to participants who had no perceived stigma (AOR = 5.07, (3.14–8.18)).

The odds of having depression among participants with hazardous alcohol use was about 2.84 times higher as compared to participants without hazardous alcohol use (AOR = 2.84, (1.32–6.09)) and the odds of having depression among participants who had currently used substances during the last three months was 1.82 times higher as compared to participants who had not currently used substances (AOR = 1.82, (1.03–3.22)) as shown below in (**Table 3**).

**Table 3:** Factors associated with depression in bivariate and multivariate logistic regression analysis among people with epilepsy at enteral Gondar zone primary public hospitals, northern part of Ethiopia (n = 556).

Explanatory variables	Depression		COR (95%CI)	AOR (95%CI)
	Present	Absent		
Marital status,				
Married	60	224	1	1
single	71	131	2.02 (1.35–3.04)	1.59 (0.88–2.87)
Divorced/widowed	41	29	5.28 (3.03–9.19)	**2.43 (1.18–4.99)** **
Living arrangement				
With family	78	290	1	1
Alone	94	94	3.72 (2.54–5.44)	1.65 (0.98–2.77)
Occupational status				
Government	13	40	1	1
Merchant	27	91	0.91 (0.43–1.95)	1.21(0.47–3.10)
Framer	52	137	1.17 (0.58–2.36)	1.31 (0.55–3.15)
Student	15	47	0.98 (0.43–2.31)	1.37 (0.45–4.14)
Household	15	38	1.23 (0.51–2.89)	1.03 (0.34–3.14)
Unemployed	50	31	4.96 (2.30–10.71)	1.41 (0.51–3.87)
Number of medications				
One	115	324	1	1
Two and above	57	60	2.68 (1.76–4.08)	**1.77 (1.02–3.09)** **
Drug Side effect Yes	34	45	1.86(1.14–3.02)	1.70 (0.91–3.19)
No	138	339	1	**1**
Frequency of seizure				
Very frequent	59	33	4.15 (2.31–7.46)	**2.68 (1.30–5.51)** **
Frequent	43	109	0.92 (0.54–1.57)	0.71 (0.37–1.37)
Occasional	36	163	0.51 (0.29–0.88)	0.53 (0.28–1.01)
Rare	34	79	1	1
Current substance use				
Yes	88	67	4.96 (3.33–7.38)	**1.82 (1.03–3.22)** **
no	84	317	1	1
Perceived stigma				
Yes	312	73	7.95 (5.31–11.91)	**5.07 (3.14–8.18)** ***
No	60	311	1	1
Hazardous Alcohol use				
Yes	56	23	7.58 (4.47–12.86)	2.84 (1.32–6.09) **
No	116	361	1	1

** = p<0.05

And

*** = p<0.001

Chi square = 11.05; DF = 8 and 0.54 = Hosmer-Lemshow test.

### Factors associated with anxiety among people with epilepsy

In the crude (bivariate logistic regression) analysis variables like living alone, being a single, being divorced/widowed, having less than or equal to 550 Ethiopian birr average monthly income, current substance use, taking two and above antiepileptic medications, 16 and above year duration of treatment, perceived stigma and hazardous alcohol use were significantly associated with anxiety. In multivariate logistic regression analysis variables including being a single, taking two and above antiepileptic medications, 16 and above year duration of treatment and perceived stigma were found having statically significant association with anxiety at a p-value less than 0.05.

In this study, the odds of having anxiety among single participants was about 1.65 times higher as compared to married participants (AOR = 1.65, (1.04–2.63)) and odds of having anxiety among respondents who had took two and above anti-epileptic medications was 2.27 times higher as compared to respondents who took only one anti-epileptic medication (AOR = 2.27, (1.42–3.62)).

The results of this study also, showed that the odds of having anxiety among participants who had perceived stigma was about 2.49 times higher as compared to participants who had no perceived stigma (AOR = 2.49, (1.63–3.82)) and the odds of having anxiety among participants with the duration of illness ≥ 16 years was 2.82 times higher as compared to participants with ≤ 5 years duration of illness (AOR = 2.68, (1.30–5.15)) as show below in (**Table 4**).

**Table 4:** Factors associated with anxiety in bivariate and multivariate logistic regression analysis among people with epilepsy at enteral Gondar zone primary public hospitals, northern part of Ethiopia (n = 556).

Explanatory variables	Anxiety		COR(95%CI)	AOR(95%CI)
	Present	Absent		
Marital status, Married	74	210	1	1
single	80	122	1.86(1.26–2.74)	**1.65 (1.04–2.63)** **
Divorced/widowed	30	40	2.13(1.24–3.66)	1.08 (058–2.01)
Living arrangement				
With family	101	267	1	1
Alone	105	83	2.09(1.45–3.02)	1.33 (0.86–2.05)
Monthly income				
≤550	66	79	1.90(1.16–3.10)	1.21 (0.69–2.15)
551–1000	54	120	1.02(0.63–1.66)	0.88 (0.51–1.50)
1001–2124	23	80	0.65(0.36–1.18)	0.66 (0.35–1.24)
>2124	41	93	1	1
Number of medications				
One	125	314	1	1
Two and above	59	58	2.56 (1.68–3.88)	**2.27 (1.42–3.62)** ***
Duration of illness				
Up to 5 years.	107	242	1	1
6–10 years.	41	80	1.16 (0.75–1.80)	1.14 (0.73–1.84)
11–15 years.	21	34	1.39 (0.78–2.52)	1.54 (0.79–3.01)
16 and above	15	16	2.12 (1.01–4.45)	2.82 (1.26–6.31) **
Current substance use				
Yes	75	80	2.51 (1.71–3.69)	1.62 (0.97–2.69)
no	109	292	1	1
Perceived stigma Yes	95	90	3.35 (2.30–3.88)	**2.49 (1.63–3.82)** ***
No	89	282	1	1
Hazardous Alcohol use				
Yes	39	40	2.23 (1.38–3.62)	1.05 (0.54–2.03)
No	145	332	1	1

** = p<0.05

And

*** = p<0.001;

Chi square = 9.06; DF = 8, and 0.42 = Hosmer-Lemshow test.

## Discussion

The current study showed that the magnitude of depression among people with epilepsy was 30.9% (95% CI, 27–35.1). This finding was in line with the study conducted in Nigeria 30.1% [17] and at central Ethiopia 32.8% [19].

However, the result of this study was lower than the study conducted in china 52.2% [10], Pakistan 60% [21], Chennai 47% [28], Benin 85.3% [29], Zambia 39.4% [20], African Togo 84% [29], and Sudan 45,5% [16]. The possible reason for the discrepancy might be the assessment tools, which was in this study we used HADS, but the study done in China was used Depression inventory for depression and general anxiety disorder -7 (GAD-7) for anxiety and Goldberg’s scale was used in African Togo and Benin. Other possible reason might be the study participants, and cultural characteristic of participant.

The magnitude of the anxiety disorders in this study was 33.1% (95% CI, 29.3–37.2).This study result was in line with the study conducted in china 33.4% [10], Nigeria 33.1% [17] and central Ethiopia 33.5% [19].

However, the finding of this study was lower than the studies conducted in Brazil 39.4% [11], Thailand 39% [9], Egypt 47% [18], Benin 84.1% and African Togo 66% [29]. The possible reason for variation may be due study participants and instrument used. The difference in study design used might be another reason for this variation. In this study, an institutional based cross-sectional study design was utilized. However, an institutional based case control study and community-based case-control study were used in Egypt and Brazil respectively.

On the other hand, the prevalence of depression and anxiety among people with epilepsy in the current study was higher than the study done in the, USA(26.9%, 25.8) [8], Canada (17.4%, 22.8%) [30], and Iran (9.5%, 24.5%) [31] respectively. The possible reason for the discrepancy might be variation in study design used, which was community-based study was used in the Canadian and Brazil but this study used an instructional based cross-section and the difference in study participants which was only among age 15–50 years and those able to read and comprehend, is included in Thailand but this study used all greater than 18years and including both those read and write and those could not read and write. Sociocultural difference might be also another possible reason for the discrepancy.

In this study, the odd of having depression was higher among divorced/widowed individuals as compared to those married. This result was supported by a study conducted in Brazil [32]. The possible justification could be, the divorced/widowed people might experience depression symptoms like feeling of hopelessness, and worthlessness due to their marital problems.

Regarding the number of antiepileptic medications, participants who had used two and above antiepileptic medications were 1.77 and 2.27 times more likely to have depression and anxiety respectively than participants those who had used one antiepileptic medication. This result was supported by study done in central Ethiopia [19, 33]. The possible justification might be due to serious adverse effect, cost of drug and drug interaction. Respondents who had experienced a seizure frequency of several times a day or shorter than seven day were 2.68 times to had depression as compared to those who had a seizure frequency occurring at interval longer than one year. This might be due to anxious and doubt about next seizure and it became lead worthlessness and feeling of hopelessness. This result was consistent to previous studies in Ethiopia, Nigeria and south India [19, 34, 35].

In this study, the current substance use has positive significant association with depression among people with epilepsy. This result was supported by the study conducted in central Ethiopia [19] and epilepsy action Australia [36]. The possible justification might be due to substance can interfere with metabolism of anti-epileptic medication, and therefore the change of seizure, some medication can enhance the toxic effect of alcohol and people can feel severely intoxicated after drinking small amount and also it might cause additional adverse effect or seizure [36].

Another factor which was associated with depression was hazardous alcohol use. Participants who had hazardous alcohol use were 2.84 times more likely to experience depression as compared to those who had no hazardous alcohol use. This result was supported by the study conducted in Germany [37]. This might be due to they might also felt depression in withdrawal state due to hopelessness, worthlessness, dysphonic feeling associated with alcohol withdrawal [38].

With respect to depression and anxiety, respondents who had perceived stigma were 5.07 and 2.49 times more likely to have depression and anxiety than those who had no perceived stigma respectively. This was supported by the study carried out in centeral ethiopia and south India [19, 39]. The possible justification might be due to the perceived stigma could predicts low self-efficacy and poor coping mechanism among people with epilepsy [40] and the affective symptoms were mostly associated with felt sigma among people with epilepsy [41].

In this particular study, long duration of illness was significantly associated with anxiety among participants with epilepsy. This might be due to those participants who had a long duration of illness become anxious about illness complication, drug adverse effect, felt sigma related illness, seizure attack and frustrated about their condition and its prospective future. However, this result was inconsistent with the study in which the authors found no significant association between anxiety and different duration of illness [42].

Besides, in this study the odds of having anxiety was higher among single participants as compared to married respondents and this result was in line with the previous study [43]. The possible justification could be that being married is a protective factor to different mental illnesses including anxiety because those married individuals can share their feelings to their couples and they can get feedback especially advice from their couples which could prevent them from developing anxiety.

## Limitations of the study

The use of retrospective items in the questionnaire may have incurred recall bias like duration of illness and duration of treatment. The cross-sectional nature of the study was its main limitation, as it cannot clarify the cause-effect relationship between outcome variables and predictive variables. Ethiopia has recognized the coronal virus infectious disease (COVID-19) case on March/13/2020; the time before this study was carried out. Since this study was carried out an instructional this might affect the result of this study.

## Conclusions

This study showed that depression and anxiety were common among people with epilepsy. Its magnitude was higher as compared to the general population. Being divorced /widowed, using two and above number of antiepileptic medications, current substance use, very frequent seizure, hazardous alcohol use, and perceived stigma were significantly associated with depression. Being single, using two and above number of antiepileptic medications, duration of illness and perceived stigma were significantly associated with anxiety. Screening, early identification and providing appropriate intervention of depression and anxiety among people with epilepsy should be great concern for the health care providers. Besides, while assessing individuals with epilepsy for depression and anxiety, giving attention to the identified above associated factors were very important.

## Supporting information

S1 Data (DTA)
